# Pain Perception Associated with Mini-Implants and Interventions for Pain Management: A Cross-Sectional Questionnaire-Based Survey

**DOI:** 10.1155/2021/4842865

**Published:** 2021-11-29

**Authors:** Swapna Sreenivasagan, Aravind Kumar Subramanian, Abirami Selvaraj, Anand Marya

**Affiliations:** ^1^Department of Orthodontics, Saveetha Dental College, Saveetha Institute of Medical and Technical Science, Saveetha University, Chennai, India; ^2^Department of Orthodontics, Faculty of Dentistry, University of Puthisastra, Phnom Penh, Cambodia

## Abstract

**Background:**

Orthodontists use mini-implants temporarily as an effective mode of skeletal anchorage devices. The placement of mini-implants can cause pain and discomfort to the patients. Patients often develop swelling, and the pain could interfere with their daily activities. Practitioners tend to prescribe antibiotics and pain medication for management.

**Objectives:**

The main objectives of this study are to evaluate the pain perception and discomfort due to mini-implant placement experienced by the patient and evaluate the interventions for pain management commonly practiced among orthodontists.

**Materials and Methods:**

The study was designed as a questionnaire-based cross-sectional study. A total of 271 patients were assessed, for whom 625 mini-implants (ranging from 1.2 to 2 mm diameter and length 8-14 mm) were placed. Pain scores were assessed using the VAS and the “Faces” pain rating scale to collect data about discomfort in daily activity and function. Data was collected from 244 patients. A total of 155 orthodontists were questioned regarding the prescription of medications and the interventions for managing pain and adverse effects.

**Results:**

Average pain score among female subjects was 16.71 and among men was 13.5. The highest pain scores were recorded for palatal mini-implants with an average score of 36.29 and the least for interradicular mini-implants with an average score of 9.02. Among the subjects, 47.9% of them took analgesics, and the most commonly prescribed analgesics were paracetamol (39%). Swelling at the site is where the mini-implants were placed, and ulceration due to implants were commonly dealt with the excision of the surrounding soft tissue, composite placement, and palliative care with oral analgesic gels.

**Conclusion:**

Female subjects had more mini-implants placed, and female subjects had also given more pain scores than their male counterparts. Palatal mini-implants caused the highest pain, followed by mini-implants placed at the infrazygomatic crest and the buccal shelf region. Palatal mini-implants caused maximum discomfort during speech and eating, followed by the mini-implant in the buccal shelf and the infrazygomatic crest region that also caused difficulty in yawning and laughing. Infiltration anesthesia was commonly given for the placement of interradicular implants and extra-alveolar mini-implants. Paracetamol was the most prescribed by the orthodontists, and more than half the doctors did not regularly prescribe antibiotics.

## 1. Introduction

One of the most significant challenges for orthodontists is to achieve successful orthodontic treatment without losing any anchorage [1]. Although numerous techniques and devices are available, TADs (temporary anchorage devices) have helped achieve appropriate anchorage control. Mini-implants are placed in various sites depending upon the demand of the case. They are of different sizes and lengths based on the site of placement and bone quality; the implants are mostly made of titanium or stainless steel. The sizes of the mini-implants range from 1.2 to 2 mm, and the length is ranging from 8 to 14 mm. Despite its advantages, it may cause pain and discomfort to the patients on its clinical use. Patients may experience pain and discomfort initially up to a week after the fixed appliances are placed. After every appointment, pain is experienced due to placement and changing of archwires and may last up to 24 hours [2, 3]. Mini-implants are mostly placed without raising any flap and are usually painless than when a flap is raised [4]. These are considered an effective mode of temporary anchorage devices and do not depend on patient compliance, but when the patient has discomfort, even adult patients often become uncooperative. Patients' compliance during orthodontic treatment depends on maintaining regular appointments, appliance care, interest, and attitude towards treatment [5].

The insertion of a mini-implant necessitates expertise and technique; slippage of the mini-implant during placement can result in soft tissue damage, which can be mitigated by utilizing a self-tapping approach, although it must still be done with caution [6, 7]. Patients also have high pain levels when drilling a pilot hole for the placement or when there are soft tissue punctures [8]. The other common cause of discomfort associated with mini-implant is seen with ulcerations which can occur as a result of soft tissue irritation in the movable mucosa; there can often be situations where the mini-implants become entrapped due to soft tissue overgrowth around the implant. This would necessitate the excision of the soft tissue to expose the implant head, which is a minor surgical operation that most patients find intolerable.

Analgesics are the primary modality to reduce pain. There is no universal or standard pain reliever. Ibuprofen, aspirin, aceclofenac, and acetaminophen are among the most commonly prescribed nonsteroidal anti-inflammatory medications (NSAIDs) [9]. These medications are known to cause side effects such as gastritis and bleeding tendencies and should be prescribed with caution. Acetaminophen/paracetamol is frequently used for orthodontic pain because it does not affect orthodontic tooth movement [10]. The intensity of pain is often diverse, and most studies prefer to employ a visual analog scale (VAS) with a rating scale to assess pain scores. The scale has a pain score recorded from 0 to 10, considering 0 as no pain and 10 is considered as unbearable pain intensity. This scale is patient-friendly, simple to interpret, and simple to use. The study was done based on the fact that there was a close connection between the remembered pain and the experienced pain, particularly for patients who had given higher scores on the VAS [11]. There has been a record of females assessing the experience of general pains such as vaccination higher than the group of males. Considering this, we evaluated the orthodontic pain associated with mini-implants in different gender, to estimate if a similar pattern followed here [12]. Dental anxiety is most common in middle-aged women; therefore, it is often essential to have a pain-free, operator-friendly, and patient comfort dental experience [13]. All stimuli are recorded as inputs from the body take a path of cyclical processing and synthesis, and these characteristic patterns are imprinted in the neuromatrix with pain and have been no different. The memory of these neurosignatory patterns is engrained in the hippocampus, which induces anxiety for the procedure and prepares the body for the prime behavioral responses of flight or fight [14].

There is a vast lacuna in literature concerning the pain and comfort of patients being treated with TADs and a lack of knowledge in managing the adverse effects. Thus, the purpose of this study is to evaluate the patient's pain perception and discomfort as a result of mini-implant insertion and the pain management strategies typically used by orthodontists. The objectives of the study were to evaluate the pain perception when using mini-implants at different sites and gender differences and how it affects the daily activities and function; to evaluate the use of anesthesia, antibiotics, and analgesic postmini-implant placement; and to evaluate the most common causes of pain and interventions by using two separate questionnaires among patients and orthodontists.

## 2. Materials and Methods

The Institutional Review Board approved the study protocol, questionnaire, and informed consent of Saveetha University. After receiving oral and written consent from patients based on the need of treatment mechanics, mini-implants were placed for the subjects. This study inserted mini-implants in the interradicular sites, infrazygomatic crest, buccal shelf, palate, and anterior midline. All of the mini-implants were manufactured by Favanchor and were made of titanium. The insertion site and indication determined the size of the mini-implant.

### 2.1. Subjects

The inclusion criteria are all subjects who reported orthodontic treatment and for whom mini-implants were placed as an adjuvant anchorage. 271 patients were enrolled in this study, and mini-implants were placed. 244 patients responded to the questionnaire, and the others refused to participate in the study. Among these, 625 mini-implants (ranging from 1.2 to 2 mm diameter and length 8-14 mm) were placed in total. This study evaluated all the mini-implants placed in various sites including the interradicular, palatal, infrazygomatic crest, and buccal shelf region. The practitioner assessing questionnaire was shared with 200 doctors. Among practicing orthodontists and postgraduate students, 155 doctors filled the questionnaire. Those who had experience with placing TADs were also questioned regarding the protocol they follow for anesthesia, the medications they prescribe, and their preferred management methods in situations of adverse effects. This study was conducted between January and July 2021.

These patients were given a self-assessment questionnaire.  Figure 1 depicts the questionnaire shared among subjects. The second questionnaire that was formulated was shared among postgraduate students or orthodontists to inquire about their experience and how they manage pain for their patients, and this questionnaire is shown in Figure 2.

### 2.2. Rating Scales

Patients' perception of pain was recorded using a questionnaire that was distributed using an online survey link. The visual analog scale was assessed using the standard 10 cm metric scale. Questions pertaining to discomfort were designed that correlate with the daily function and activities of the patient. These questions were answered using the Wong-Baker Faces Pain Rating Scale. VAS score was used to assess the pain and swelling. The patient's daily activity could be effectively affected, and the factors we took into consideration were leisure, speech, ability to eat hard and soft food, drinking, laughing, and yawning. These questions were given a score rating of 0-5, given that 0 meaning no discomfort to 5 indicating worst pain. Patients were also questioned about their use of pain medication postplacement of mini-implants. No patient answered the questionnaire more than 1 month after the mini-implant was placed.

The orthodontists were questioned regarding the prescription of antibiotics and pain medication after the placement of TADs; they were also questioned regarding the adverse effects of swelling, soft tissue entrapment, and their call for management. Local anesthesia is used by topical application, infiltration, or via block for placement of mini-implants. The need and the preferred route of administration was asked. Despite administration, patients often tend to experience pain during the mini-implant placement or the driver's detachment from the head of the implant postplacement.

The data thus collected were used to assess the pain and discomfort of the patients as well as the management options for pain and other side effects experienced after mini-implant placement.

### 2.3. Statistical Analysis

The statistical analysis was done using the IBM SPSS statistics 20 software. Descriptive statistics were evaluated for the orthodontists who answered the questionnaire and the subjects for whom mini-implants were placed. Graphs were obtained based on the VAS pain scores and Faces pain scores.

## 3. Results

### 3.1. Descriptive Statistics (Table 1)

#### 3.1.1. Self-Report Questionnaire from Patients

The questionnaire was collected from 244 subjects who underwent treatment with mini-implants. The patients who did not complete the questionnaire were excluded from further analysis. For 75% of the patients, interradicular mini-implants were placed, 12% had implants placed at the IZC, 9% had implants placed in the buccal shelf, and 8.5% of patients had mini-implants placed in the palate. The mean age of the patients was 23.9 ± 6.4 years, with 156 females and 88 males consenting.

#### 3.1.2. Practitioner Assessment Questionnaire

The questionnaire was circulated among 200 orthodontists, and 155 filled it. The mean age group of the orthodontists was 30 ± 6 years, 83 were female, and 71 were male; 90 of them were postgraduate students, and 64 were practicing orthodontists. 124 doctors had an experience of fewer than 5 years, 12 doctors between 5 and 10 years, 10 of them with an experience of 15 years, and 8 of them more than 15 years.

*(1) Pain Perception of Patients*. The pain score was evaluated for a score of 70, and the highest score recorded was 49, and the minimum score was 0. The maximum pain recorded was 49 for palatal mini-implants.

*(2) Gender Differences*. More female patients reported orthodontic treatment, and more female patients were treated with temporary anchorage devices. Among them, the female patients had stated an average pain score of 16.71, and on average, the pain score among male patients was 13.5 (Figure 3).

*(3) Type of Implant*. The average pain score for the implant placed at the infrazygomatic crest was 31.8, at the buccal shelf was 30.35, and at in the palate was 36.29, whereas the interradicular mini-implants had an average pain score of 9.02. This suggested that the implants placed in the extra-alveolar site almost had aching pain, but no pain to mild pain was only present in the case of interradicular mini-implant (Figure 4).

*(4) Daily Activities and Function*. In Table 2 and Figure 5, the questions regarding daily activities were assessed using the Faces scale where 0 indicated no hurt and 5 indicated hurts worst. All the extra-alveolar screws had scored more than 2 and affected leisure activities. The speech was highly affected in the palatal implant (score of 2.82) followed by the buccal shelf (score of 2.57) and infrazgyomatic crest (1.8). The pain scores for taking a big bite and eating hard food were maximum for the buccal shelf (2.17) and palatal mini-implant (3.86). Overall, the maximum difficulty with eating was due to the mini-implants placed at the IZC followed by palatal mini-implants (score of 2.17), and the buccal shelf score was 1.17. The scores for difficulty in laughing had the maximum discomfort in the buccal shelf (3.05) followed by at the IZC region 2.8 and a score of 2.57 for mini-implants in the palate. On assessing all the questionnaires pertaining to mini-implants, the interradicular mini-implants all had scores less than 2. This suggested that they did not cause any discomfort or pain that affected daily activities and functions.

On questioning, if the patient skipped work after being placed with mini-implants, 72% did not take any break from work. Among those who missed work, 44% of them missed work for one day, whereas few took leave from work up to 3-7 days. 77.4% of subjects did not have any difficulties in continuing their leisure activities. 29.5% of patients reported having disturbed sleep postimplant placement.

*(5) Use of Anesthesia for Mini-Implant Placement*. All the orthodontists confirmed that local anesthesia is needed to place mini-implants. For placement of interradicular mini-implants, 82% of doctors gave infiltration, 14.9% said only topical anesthesia would be sufficient, and very few doctors gave a nerve block. In order to place extra-alveolar screws at the infrazygomatic crest, buccal shelf, or the ramus, the requirement of a nerve block was suggested by 48.5% of the doctors, and 51.5% of doctors felt that infiltration of the local anesthetic would be sufficient. 30% of the patients complained of pain despite the anesthesia, and 20% reported having discomfort during detachment of the driver after the implant was placed. The majority of them did not have any pain during placement.

*(6) Most Common Cause of Pain as Reported by Practitioners*. The most common cause of pain as reported by orthodontists is that their patients reported pain at the site of insertion (35%) followed by ulceration caused due to implant (28%). The lesser common causes that caused pain to the patient were incorrect placement (14%) and infection (13%). Few patients had reported pain and discomfort due to difficulty in eating and swelling (4%).

*(7) Specific Hygiene Instructions to Patients*. The majority of the doctors had advised the use of mouth-rinse postplacement. Some had suggested that mouth rinse was done with chlorhexidine, while others had suggested salt in lukewarm water. Few doctors suggested cleaning the implant head with a soft toothbrush or ear bud dipped with chlorhexidine and, most importantly, preventing any food accumulation.

*(8) Use of Antibiotics and Analgesics*. When the patients were asked if they took analgesics after the placement of mini-implants, 47.9% of the patients had used analgesics. According to the patients, the most common drug prescribed to them was paracetamol (39%) followed by aceclofenac (11%) and ibuprofen (7%). Most of the patients did not recall the drug they had taken (43%).

57% of the doctors had reported that they do not prescribe antibiotics after mini-implant placement, but the remaining 43% gave antibiotics routinely after the placement. 14 doctors did not specify what antibiotics they prescribed. Amoxicillin was the most commonly prescribed, followed by ciprofloxacin. 70% of the doctors routinely prescribed analgesics. The most commonly prescribed NSAID was paracetamol or acetaminophen (80%), followed by ibuprofen and aceclofenac.

*(9) Intervention and Management for Pain*. 48% of doctors said they did not observe any swelling or soft tissue overgrowth where the mini-implants were placed, whereas 52% reported soft tissue overgrowth. The most common intervention during soft tissue swelling that the practitioners did was to remove and reposition the implant as suggested by 60% of the doctors. The second most common intervention was to excise the soft tissue, followed by assessing the situation. Most of the doctors had observed ulceration only sometimes (59%), 10 doctors had reported they observed ulceration very often, and 25% had never observed their patient developing any ulcer. When the patient developed an ulcer, 54% of the doctors wanted to place composite on the head of the screw, to prevent repeated soft tissue overgrowth, 49% gave oral ulcer gels either alone or as an adjuvant, and 25% of practitioners gave palliative care with placement of wax on the implant head.

## 4. Discussion

Pain is a subjective phenomenon and often is tedious to assess and depends on various variables. It tends to vary based on gender, age, the site of mini-implant placement, and the subject's previous experience of pain [15]. In our study, female subjects gave a higher pain score.

The scores for pain in our were relatively lesser for interradicular mini-implant with an average of 9.02. In a randomized trial conducted by Ganzer et al., it was pointed out that there was pain and discomfort associated with the placement of mini-implants, but this pain was lesser in intensity in comparison to postoperative pain following tooth extraction [16]. On comparing the pain of mini-implant placement to initial tooth alignment, the mini-implant procedure caused less pain [17]. In a pilot study by Brandão et al., they had pointed out a ready acceptance to mini-implants observed in 90% of the patients and 50% had no discomfort and that patients adapted to mini-implants within 3 days [18].

We observed a high pain score in the palatal region (36.29) followed by the mini-implants placed in the infrazygomatic crest region (31.8) and at the buccal shelf (30.35). The mini-implant placement in this region often requires a higher torque value due to the higher bone density and often experiences high levels of pain immediately postplacement [19]. In a cohort study, researchers had pointed out that the buccal placement of mini-implants is more painful than it finally is [8]. Kuroda et al. reported that mini-implant placement in the IZC region and found a decrease in VAS score from 1-day postplacement to the 7th day. The highest VAS score in this study was reached 1-hour postplacement [4]. The variation in the design of the mini-implant has no role in the postinsertion pain levels [20]. Kawaguchi et al. had compared the pain perception using VAS scores in buccal and palatal miniscrews and the miniplates. The highest pain scores were recorded for miniplates. Miniscrews are preferable over miniplates as a choice when patient discomfort is considered [21]. When the buccal miniscrews are placed without flap, there is a minimal report of pain and swelling [22]. Pain intensity in the palate and tongue is higher in skeletal anchorage devices when compared to a transpalatal arch [23].

Du et al. had compared in a study the pain in microimplants, mini-implant, and miniplates. They had recorded a VAS score of 61.1 mm. They had observed a high VAS score when a palatal mini-implant was placed due to irritation to the tongue [24]. The highest score for pain and discomfort affecting the daily activities and function was observed for the palatal mini-implants in our study. Patients had expressed difficulty in speech and eating. We also observed that the mini-implants placed at the buccal shelf and the infrazygomatic crest had caused discomfort during laughing, yawning, and eating.

Most of the orthodontists we questioned preferred the use of infiltration anesthesia before the placement of the mini-implant. It is not uncommon for certain practitioners to place mini-implants by merely using topical anesthesia. Patients are often anxious about the injection [13]. Local anesthesia is injected often via infiltration. However, Kwong et al. had suggested that the numbing effect on the gingiva and, to some effect, the periosteum will be helpful, but when the interradicular implants are placed, complete numbing of the gingiva, periosteum, and the cortical plate are required, hence an infiltration [25]. In a randomized trial comparing a compound topical anesthetic to a needle administered anesthesia, participants who received only topical anesthesia had more pain and more anesthetic failures than those given injected anesthesia [26]. In yet other studies point out that topical and infiltration anesthesia were compared for mini-implant placement. The most unpleasant sensation that patients endured during the placement was the pressure during placement. Also, patients for whom topical anesthesia was given before placement developed more pain [27, 28].

Maintenance of utmost sterilization protocol is essential in order to prevent infection, and more than half the doctors do not recommend the use of antibiotics postplacement. Patients are also instructed to regularly use mouth rinse and clean the surface of the implant head in order to prevent the accumulation of plaque that can lead to inflammation and infection. In contrast, most practitioners readily prescribed analgesics, and paracetamol was the most commonly prescribed drug. Ibuprofen, acetaminophen, and aspirin are often used in relieving orthodontic pain. These are also commonly prescribed after placement of mini-implant [29, 30]. Anesthetic gels are often prescribed when irritation from band wire occurs and often makes it painless [31]. For adverse effects like swelling and soft tissue growth, effective management can be done with repositioning the implant, excision of the soft tissue overgrowth, and placement of soft material like composite on the implant head, which will also prevent ulceration. Oral analgesics are often prescribed for palliative care and pain relief caused by ulceration of the implant head.

The limitations of this study are as follows: the questionnaire was not given at a set interval, and most of the previous studies had shown that the maximum VAS scores were recorded between 1 and 6 hrs after insertion of the mini-implant. There is a reduction of pain after about 1-week postplacement of the mini-implant [21]. Our study did not evaluate the pain-related factors associated with the placement of mini-plates. Prolonged discomfort was observed for palatal miniscrews rather than the buccal.

## 5. Conclusions

Practitioners should be aware of the discomforts experienced by their patients in order to achieve maximal treatment efficacy and happy compliant patients. During placement of mini-implants, female patients reported more pain. The mini-implants placed in the palatal, infrazygomatic crest, and the buccal shelf region reported high pain scores and affected daily functions. Analgesics should be prescribed to ensure pain-free treatment with TADs. Proper placement techniques and effective palliative care should be utilized to prevent the development of ulceration, soft tissue enlargement, and swelling.

## Figures and Tables

**Figure 1:** Self-report questionnaire concerning pain and discomfort.

**Figure 2:** Practitioner assessment questionnaire for pain and discomfort associated with TAD placement.

**Figure 3:** Pain scores based on gender.

**Figure 4:** Pain scores based on type of mini-implant.

**Figure 5:** Comparison of discomfort in various activities among different types of implants.

**Table 1:** Descriptive statistics.

Subjects who received mini-implants	88 male	156 female	Mean age: 23.9 ± 6.4 years
Mini-implants placed based on location (percentage)			
Interradicular	75%		
IZC	12%		
Buccal shelf	9%		
Palatal	8.5%		
Orthodontists who answered the question	71 male	83 female	Mean age: 30 ± 6 years
Years of experience (No. of doctors)			
Less than 5 years	124		
5-10 years	12		
10-15 years	10		
> than 15 years	8		

**Table 2:** Discomfort in daily activities.

Question	Number of subject who answered “yes”	Number of subject who answered “no”
Staying away from work postinsertion of implant	66	177
Staying away from leisure activities	54	189
Sleep disturbance due to pain	72	171
Have you taken analgesic postmini-implant placement procedure	117	126

## Data Availability

Any data related to the study can be provided on reasonable request.
